The article "Improving the Survival Time of Multiagents in Social Dilemmas through Neurotransmitter-Based Deep Q-Learning Model of Emotions" was published in 2022. Journal: J Healthc Eng.

# Improving the Survival Time of Multiagents in Social Dilemmas through Neurotransmitter-Based Deep Q-Learning Model of Emotions

**DOI:** 10.1155/2022/3449433

**Published:** 2022-01-25

**Authors:** Awais Hassan, Maida Shahid, Faisal Hayat, Jehangir Arshad, Mujtaba Hussain Jaffery, Ateeq Ur Rehman, Kalim Ullah, Seada Hussen, Habib Hamam

**Affiliations:** ^1^Department of Computer Science, University of Engineering and Technology, Lahore 54890, Pakistan; ^2^Department of Computer Engineering, University of Engineering and Technology, Lahore 54890, Pakistan; ^3^Department of Electrical & Computer Engineering, COMSATS University Islamabad, Lahore Campus, Lahore 54000, Pakistan; ^4^Department of Electrical Engineering, Government College University, Lahore 54000, Pakistan; ^5^Department of Zoology, Kohat University of Science and Technology, Kohat, Khyber Pakhtunkhwa, Pakistan; ^6^School of Electrical and Computer Engineering, Haramaya Institute of Technology, 138 Diredawa, Ethiopia; ^7^Faculty of Engineering, Uni de Moncton, Moncton NB E1A3E9, Canada; ^8^Spectrum of Knowledge Production & Skills Development, Sfax 3027, Tunisia; ^9^School of Electrical Engineering, Department of Electrical and Electronic Engineering Science, University of Johannesburg, Johannesburg 2006, South Africa

## Abstract

In multiagent systems, social dilemmas often arise whenever there is a competition over the limited resources. The major challenge is to establish cooperation among intelligent virtual agents for solving the situations of social dilemmas. In humans, personality and emotions are the primary factors that lead them toward a cooperative environment. To make agents cooperate, they have to become more like humans, that is, believable. Therefore, we hypothesize that emotions according to the personality give birth to believability, and if believability is introduced into agents through emotions, it improves their survival rate in social dilemma situations. The existing researches have introduced different computational models to introduce emotions in virtual agents, but they lack emotions through neurotransmitters. We have proposed a neurotransmitters-based deep Q-learning computational model in multiagents that is a suitable choice for emotion modeling and, hence, believability. The proposed model regulates the agents' emotions by controlling the virtual neurotransmitters (dopamine and oxytocin) according to the agent's personality. The personality of the agent is introduced using OCEAN model. To evaluate the proposed system, we simulated a survival scenario with limited food resources in different experiments. These experiments vary the number of selfish agents (higher neuroticism personality trait) and the selfless agents (higher agreeableness personality trait). Experimental results show that by adding the selfless agents in the scenario, the agents develop cooperation, and their collective survival time increases. Thus, to resolve the social dilemma problems in virtual agents, we can make agents believable through the proposed neurotransmitter-based emotional model. This proposed work may help in developing nonplayer characters (NPCs) in games.

## 1. Introduction

Artificially intelligent agents are being employed in the field of robotics [1], games [2], entertainment [3], education [4], healthcare [5], customer services [6], and many more. A multiagent system (MAS) is a group of autonomous agents interacting in the same environment to achieve a common goal [7]. In these multiagent systems (MASs), situation of social dilemmas often arises. As Shaver [8] defined, social dilemmas mean that individuals from a group, society, or culture compete to use limited public goods [9] shared among them. The case of social dilemmas occur in many computational problems such as in competitive structure during file sharing in peer-to-peer systems [10], limited food resources, and their high consumption during simulated survival scenarios [11] and common shared medium among all nodes during bandwidth allocation in telecommunication systems [12].

The capacity to solve social dilemma problems benefits the whole community in the long run. For instance, in Hardin's “Tragedy of the Commons” [13], a social dilemma in the survival scenario, a common pasture, is shared among a community of herdsmen to graze sheep. If each herdsman has a small number of sheep, then the pasture provides plenty of grass to the animals of all herdsmen, which is beneficial for the community in the long run. However, if each herdsman increases his number of sheep for his benefit, the grass is soon scarce in the pasture. The literature suggests that cooperation is necessary among the people to resolve social dilemmas [14–16]. Therefore, to solve the social dilemma among AI-controlled virtual agents, these agents must have believability so that cooperation and coordination are developed among them [17].

The general idea of believability in virtual agents is realistic and human-like characters in virtual worlds. Bogdanovych et al. [18] define a believable virtual agent that is an autonomous agent with its behavior, personality, distinct emotional state, internal goals, and beliefs. This definition explains that personality, emotions, motivation, and social relationships are the key features of believable agents. It suggests that intelligent agents can effectively deal with social dilemma problems when equipped with an empathetic personality through positive emotions, internal motivations, and the capacity to alter their decisions after observing the environment and needs of other agents.

In the literature, believability has been explored initially for virtual agents but only limited to their visual appearance [19]. These works focused on facial expressions [20], motion control [21], hair [22], and dress [23] simulation of virtual agents. Later, many researchers argued that only the physical properties of agents are not sufficient to introduce believability, which can be introduced by making agents rationale that makes goal-oriented decisions [10]. Therefore, the focus was shifted towards the development of models for utility-maximizing rational agents [24].

The rational agents are not adaptable in complex environments as they tend to make self-centered decisions [25]. Hence, these agents must be equipped with emotions, as emotions can affect their goals [26], which in turn alter their actions, thus playing a vital part in decision-making capabilities. The neurological studies suggest that an emotional mind has a substantial contribution to the process of decision-making [27]. Therefore, emotions are a necessity to be included in the rational reactive models for the creation of believable artificial intelligent agents [25]. Literature also suggests that person-specific elements, such as personality [28, 29] and mood [30], also affect the emotion processing mechanism. Therefore, it is also necessary to model the effect of personality on the emotion processing mechanism for the creation of believable virtual agents.

In the last decade, there has been a tremendous advancement in affective computing by introducing various emotional models [31–39] for virtual agents, but these models fail during social dilemmas scenarios. In our opinion, without cooperation between artificial intelligent agents, all the agents' survival as a community is impossible. However, simple rule-based emotions are not enough for multiagents while considering the community's collective survival [38]. Neurotransmitters are the chemicals that control emotions in humans. The development of virtual neurotransmitters in intelligent agents can regulate emotions and help improve the agents' decision-making capabilities. We argue that a neurotransmitter-based emotion modeling in intelligent agents can introduce cooperation and coordination among multiagents and provide collective survival of the community in a virtual world. More specifically, this paper addresses the following research questions.

- How do emotions introduce believability in virtual agents?
- How do emotions increase cooperation between agents?
- Does the introduction of emotions by controlling and regulating the virtual neurotransmitters improve the decision-making capability of agents?

The major contribution of this paper is the neurotransmitter-based deep Q-learning model for emotional modeling in virtual agents. According to the OCEAN model, a selfless and selfish personality in virtual agents is established through agreeableness and neuroticism personality traits. Believability based on emotion regulation through dopamine and oxytocin is introduced specifically to the personality of the agent. For the solution of social dilemmas in survival scenario of multiagents, cooperation is established among the agents using the proposed neurotransmitter-based deep Q-learning model.

We have tested the proposed model through simulation performed in a grid world environment developed in the Unity3D platform. Experimentation is conducted by varying the number of selfless and selfish agents, and agents learn to keep their neurotransmitters in the desired range according to their personality. The agents achieve maximum reward by performing the specific actions that best suit their personality. When we increase the number of selfless agents with a high agreeableness personality trait, they start cooperating with others by regulating their positive emotions through neurotransmitters according to their personality, resulting in improved social dilemmas.

The rest of the paper is structured as follows.  Section 2 provides a detailed literature survey of the previous work done in this domain.  Section 3 presents the proposed solution discussing the model's architecture philosophy and the working of emotional agent in the environment.  Section 4 describes the experimentation for the evaluation of the proposed solution. Sections 5 and 6 consist of Results and Discussion.  Section 7 concludes the paper.

## 2. Related Studies

### 2.1. History of Emotional Models for Believable Agents

The field of emotion-based believable virtual agents flourished after the research works of Bates [40] and his students [41]. They built emotional agents for the Oz project equipped with reactive capabilities and memory. Moreover, they were also introduced with social relationships and emotions models based on Ortony, Clore, and Collins's (OCC) theory of emotions [42]. The research only focused on the agents from an artistic point of view (i.e., appearance-based). The impact of the believable agent's internal and external motivation on its emotions and behavior was not considered. Sloman [43] tried to remove the deficiencies in Bate's Model by introducing a “broad” emotion model. He presented a design-based approach to develop intelligent and motivated agents. While conducting further research to develop a more flexible architecture for autonomous agents, Sloman developed a toolkit named SIM_AGENT [44] for agent development. Many interactive mechanisms of agents, that is, processing different motives, choosing a motive according to the situation, and then acting on it, were included in that toolkit.

For the simulation of dogs and other creatures, an autonomous architecture for agents was proposed by Blumberg [45]. The agents' behavior was created as independent objects, and a specific behavior was achieved by switching between the agent's goals. Hence, the agent would be in a single emotional state at a time, but this architecture failed to address Ekman's complex, compelling, and comprehensive behavioral model [46].

Cathexis is a computational emotional model for producing emotions and their control on agents' behavior proposed by Velàsquez et al. [47]. Although, this model integrated both cognitive and noncognitive promoters of emotions, it did not consider the impact of personality on the emotional changes. However, this model opened new and versatile paths for implementing emotions in agents.

Loyall [48] recognized that personality and emotions both are necessary for the creation of believable agents. He suggested that extensive computations for introducing emotions must also be believable. El-Nasr et al. [49] proposed PETEEI (pet with evolving emotional intelligence). This architecture models the behavior of pet dog through reinforcement learning. This model provided the agent with a feedback mechanism that allowed the agent to adapt its behavior after learning from its experiences.

In the same way, El-Nasr et al. [34] also presented the model FLAME (Fuzzy Logic Adaptive Model of Emotion). This model was also based on the Ortony, Clore, and Collins's (OCC) theory on emotions. An inductive learning system was used to find the hidden patterns in events and connections among objects. Emotions were created based on the appraisal of events according to the fuzzy rules. This model was a significant step forward in determining how emotions change the behavior of agents. Both PETEEI and FLAME were designed for virtual pets; therefore, personality was not included in these models.

Moreover, to improve military simulations, believability in autonomous virtual human agents has also been explored. For this, Silverman et al. [50] compiled human behavior models (HBMs)/performance moderator functions (PMFs), which filtered hundreds of human behavior models helpful in the implementation of behavioral models for believable virtual humans.

Silverman et al. [51] and Silverman, Johns, et al. [52] presented a model that focused on the effects of cognition, stress, perception, and social processes on emotions and virtual decision-making agents. Moreover, they also explored various methods for implementing existing behavioral models in game engines.

Recently, Yang et al. [53] extended the models proposed by Silverman et al. [51] and Silverman, Johns, et al. [52] by introducing the social learning component. This extended model facilitated learning the relationships between agents. Thus, the decision-making capabilities of virtual agents were improved using this information. In the same way, You and Katchabaw [54] presented a model that helped integrate the different psycho-social models.

### 2.2. Introduction of Cooperation and Emotions through Reinforcement Learning

Diallo et al. [55] proposed that deep reinforcement learning algorithms can be used to cooperate between two agents to achieve a specific task. The fully observable ping-pong scenario tested different deep reinforcement learning algorithms by teaming up the two agents to play against the hard-coded player. Results showed that deep Q-network with double Q-learning gave the best results in the ping-pong scenario by maximizing the total reward of two agents. Cooperation was achieved to some extent, but there was no communication between the agents.

Broekens et al. [56] proposed an emotional model of joy, distress, hope, and fear using reinforcement learning for a single agent in the maze scenario. They mapped the RL primitives to these four emotions. Fear and hope were mapped to the values of the states, whereas joy and distress were mapped to the error function. They hypothesized that for adaptive behavior learning, agents must have complex emotional feedback from the environment. Experiments were done on a maze scenario simulated in JAVA. The results showed that the function of emotion is useful for the adaptive behavior of the agent.

Sequeira et al. [57] proposed an intrinsically motivated reinforcement learning framework to overcome the agent's perceptual limitation by implicitly encoding the information. Reward functions were evolved through the fitness function of genetic programming, and the best-suited functions were adopted to maximize the reward. Many experiments were done on the grid world foraging environment and Pacman scenarios. Results showed that emotional appraisal signals improved the decision-making capability of the agent.

### 2.3. Introduction of Cooperation for Handling Social Dilemma in Agents

Introducing cooperative behaviors among multiagents has been a topic of interest among researchers for solving social dilemmas. Researchers have investigated the introduction of emotions among two agents for establishing cooperation in social dilemma scenarios [11, 58, 59].

Yu et al. [58] proposed a double-layered framework with emotional multiagent reinforcement learning that provided agents with emotional and cognition capabilities to induce cooperation. Intrinsic rewards were used to learn the inner layer of the framework, where one emotion emerges as a dominant factor from the emotional processes of the agent. In the outer layer of the framework, the emergent emotion was used as biased reinforcement signals to learn the related cognition and behavioral changes. Experimental results showed that the agent's heterogeneities and different network topologies also had a noteworthy impact on the learning behaviors of the agent.

Huang et al. [59] modeled a dynamic network whose weights evolve with the game's strategy for modeling the effect of cooperation. The hypothesis was that different agents perceive the puzzle of social dilemmas differently. Tests were conducted on two spatial games (prisoner's dilemma and snowdrift game). According to the results, for a small temptation to defect in the game, high network evolution strength was needed for cooperation. The vice versa was also correct.

Leibo et al. [11] introduced sequential social dilemmas to analyze the dynamics of agents' learning policies using deep Q-network. Previously, in Matrix games like the prisoner's dilemma choice to defect or cooperate was treated as a single action. However, in social dilemmas of the real-world, cooperation can be learned after devising the whole policy. For this, the authors tested their hypothesis on two games (fruit gathering and wolf pack hunting game). The experimental results showed that cooperative policies were easier to learn in the fruit-gathering game than wolf pack hunting. As in the wolf pack hunting game, a lot of coordination was needed for learning the cooperative policy. In this research, the personality and emotions of the agents were not taken into account.

A research matrix for comparison of related works is presented in Table 1, where we categorized the existing works on the basis of reinforcement learning, social dilemma in MAS, use of emotions in social dilemmas, and cooperation of multiagents.

## 3. Proposed Methodology

### 3.1. Architecture Philosophy

The proposed solution is based on the philosophy shown in Figure 1.

In humans, neurotransmitters are called chemical messengers in the brain. Different levels of these neurochemicals control emotions. However, what emotion has to be expressed depends on the specific personality of humans. Similarly, by varying the levels of virtual neurotransmitters in agents, particular emotions can be acquired according to the agents' personalities. These personality-specific emotions will lead to believability in virtual agents, which is necessary to solve social dilemmas with limited resources.

### 3.2. Working of Agent in Environment

The model's architecture diagram (Figure 2) is inspired by Barto et al. [29] concept of extrinsic and intrinsic motivation of agents in reinforcement learning.

According to the architecture diagram (Figure 2), the emotional agent can observe the environment. After receiving the knowledge of the environment, the agent performs specific actions in the environment and its state changes. On performing these actions, the agent receives some reward according to extrinsic and intrinsic motivation based on the agent's state. The cumulative reward is calculated by combining rewards based on extrinsic and intrinsic motivation. This cumulated reward is also fed into the agent's brain, along with the state of the environment. The brain processes this information and decides the best action for the agent to take in the environment. This process continues, and the agent tries to maximize its reward by performing the best actions in the environment.

### 3.3. Emotional Agent

#### 3.3.1. Emotional Agent

The environment is a fully observable grid world consisting of certain virtual agents with different personalities and food reservoirs to gather food. Information about the environment is passed to the brain of the agent in the form of state space. The state-space consists of the location of all food reservoirs, available food in these reservoirs, the total number of alive agents in the environment, the position of these agents, the food level of all these agents, and time passed in the environment. Agent's internal information, that is, its food level and the levels of its neurotransmitters, are also a part of state space.

#### 3.3.2. AGENT Actions

Every agent is allowed certain specific actions that it can perform in the environment. With the actions of up, down, right, and left, it can move in the environment or stay in its position by not act. It can also eat from the food reservoir and share food with the other agents. In short, an agent can perform any one of the total 7 actions available in the action list. The action list is{No action, Up, Down, Left, Right, Eat, and Share}.

#### 3.3.3. Rewards System Based on Extrinsic Motivation

In reinforcement learning, there are two types of rewards.

- Rewards based on extrinsic motivation
- Rewards based on intrinsic motivation

Psychologists have distinguished between extrinsic and intrinsic motivation. Extrinsic motivation is defined as propelling us to do a task based on some particular rewarding outcome. Whereas intrinsic motivation drives us to do a job because it is inherently enjoyable. In short, behavior driven by external reward is extrinsic motivation, whereas the behavior driven by internal reward is intrinsic motivation. Extrinsic motivation arises after observing the rewards present in the environment. Intrinsic motivation of the human emerges from the person's personality [60] and neural networks and dopaminergic systems present in the person's brain [61]. Hence, for the intrinsic motivation in the agent, it is necessary to introduce virtual personality and emotions by controlling the neurotransmitters or brain chemicals in the agent.

#### 3.3.4. Rewards System Based on Intrinsic Motivation

Intrinsic motivations of the agents are inspired by the drive theory of Hull in psychology [62–64]. The specific personality of the agent has some particular emotions. These emotions are achieved by balancing and controlling the neurotransmitters. This balancing of neurotransmitters drives the agent to perform the specific actions related to the agent's personality.

#### 3.3.5. Personality

The personality of the agents is based on the OCEAN model (Figure 3), also known as the Five-Factor Model (FFM) developed by Robert McCrae and Paul Costa [65]. The OCEAN Model consists of big five personality traits: Openness, Conscientiousness, Extraversion, Agreeableness, and Neuroticism.

Openness is an extensive realization of diversity of experience, exceptional ideas, and curiosity. Open to experience, people are willing to seek and strive for new things and are curious intellectually.

Conscientiousness is the likelihood of a person to be dutiful, self-disciplined, and goal-oriented against all measures. It can be associated with how people direct, regulate, and control their stimulus responses.

Extraversion is related to extrovert, action-oriented, and enthusiastic people interacting and engaging with external people and the outside world. The personality trait of agreeableness is marked with kind, considerate, helpful, trustworthy, and generous nature. Agreeable people have a significant concern for social peace, and they have an optimistic perspective of humans. Selfless people fall under this category. Neuroticism is marked with people having negative emotions such as depression, anger, and anxiety. Ordinary situations and minor frustrations are threatening and hopelessly tricky for them. The occurrence of this trait is most likely to make a person selfish.

#### 3.3.6. THE Proposed Personality Model

Studies suggest that people having a high level of Neuroticism and low level of Agreeableness are usually selfish and self-centered [66]. However, people having a high level of Agreeableness and low level of Neuroticism are generally selfless and empathetic [67]. As this paper deals with the social dilemma situation, only those personality traits are required that are most likely to make the agents selfish or selfless. Hence, the personality of Agreeableness and Neuroticism is considered from the OCEAN Model for the emotional agents. These personality trait values remain within the range of [0, 1].

#### 3.3.7. Neurotransmitters

The emotional chemicals involved in the Limbic System [61] are used to determine the agents' emotions. The basic four emotional chemicals (Figure 4) are dopamine, serotonin, oxytocin, and endorphin [68].

The neurotransmitter that is related to motivation and reward chemical is dopamine. It is released by a small portion of the brain, hypothalamus, located at the base of the brain. Drive, focus, memory, and attention are associated with this chemical.

Serotonin is the neurotransmitter known as the happiness hormone. Mood upliftment and relaxation are achieved by the correct portion of the serotonin level in the body. Hypothalamus also generates the bonding hormone known as oxytocin. Social behavior and feelings of calmness and contentment are related to this neurotransmitter. In pain, stress, and fear, endorphins are the neurotransmitters released. These allow us to cope with the pain.

In his book [69], Simon Sinek categorized dopamine and endorphin as selfish chemicals, whereas oxytocin and serotonin as selfless chemicals. For the situation of social dilemma in virtual agents, dopamine and oxytocin from each category are considered. Neurotransmitters are maintained within [0,10], with 0 as the lowest level and 10 as the highest level. This paper shows that high level of virtual oxytocin creates the emotion of love, empathy, and selflessness among agents. Low levels of oxytocin generate the emotions of selfishness. Dopamine represents the motivation and goal achievement chemical.

#### 3.3.8. Neurotransmitters to Agents Action's Mapping

As mentioned earlier, the agent can perform any action available in the action list at a time step. While doing these actions, the level of neurotransmitters within the agent changes. For example, if the agent is hungry and takes those movement actions that will reduce its distance from the reservoir, its dopamine level increases. This level of increase depends on the distance between the agent and the food reservoir. Dopamine level increases more speedily if the specific action makes the agent closer to the reservoir. But this level decreases if some action makes the agent move away from the food reservoir. Since during the movement, the agent does not interact and share food with the other agents; therefore, its level of oxytocin decreases. When an agent performs the eat action, the dopamine level increases more swiftly as it has achieved its goal, but the level of oxytocin remains the same at that time. When the agent performs the share action, both the level of dopamine and oxytocin increase. It is because the agent is performing a selfless action.

#### 3.3.9. Extrinsic Motivation

Every agent has a certain food level, and the agent dies if the food level reaches 0. Since the goal of this research is the collective survival of agents; therefore, extrinsic motivation for the agents is the aliveness of every agent. Thus, extrinsic motivation drives the agent to take actions for the survival of all the virtual agents.

#### 3.3.10. Reward Calculation

According to the value of agreeableness and neuroticism, the agent can have different percentages of selflessness and selfishness in its personality as shown in Table 2. In this model, the selfless agent has the agreeableness of 0.8% and 0.2% of neuroticism. Vice versa is correct for the selfish agent.

As already explained, a high level of virtual dopamine and oxytocin creates the emotion of love, empathy, and selflessness among agents. A low level of oxytocin generates the emotions of selfishness. The emotional state of the agents is shown by the following two functions given below:

(1) $$\begin{array}{c} F_{\text{SL}}\left(\text{Dop},\text{Oxy}\right)=\text{sgn}\left(\frac{\left|\left(\left(\text{Dop}/4\right)-1\right)\right|+\left(\left(\text{Dop}/4\right)-1\right)}{2}\right)*\text{sgn}\left(\frac{\left|\left(\left(\text{Oxy}/5\right)-1\right)\right|+\left(\left(\text{Oxy}/5\right)-1\right)}{2}\right),\\ F_{\text{SF}}\left(\text{Dop},\text{Oxy}\right)=\text{sgn}\left(\frac{\left|\left(\left(\text{Dop}/2\right)-1\right)\right|+\left(\left(\text{Dop}/2\right)-1\right)}{2}\right)*\text{sgn}\left(\frac{\left|\left(1-\left(\text{Oxy}/4\right)\right)\right|+\left(1-\left(\text{Oxy}/4\right)\right)}{2}\right), \end{array}$$

where subscript SL represents the Selfless and SF represents the Selfish. Sgn is the signum function, and abs is the absolute function. *F*_SL_(Dop, Oxy) only returns true when the neurotransmitters have reached the specific level, that is, dopamine > 4 and oxytocin > 5. *F*_SF_(Dop, Oxy) returns true only when dopamine > 2 and oxytocin < 4.

Reward based on the intrinsic motivation *R*_Int_ is given as follows:

(2) $$\begin{array}{c} R_{\text{Int}}=\text{Value of agreeableness}*F_{\text{SL}}\left(\text{Dop},\text{Oxy}\right)+\text{Value of neuroticism}*F_{\text{SF}}\left(\text{Dop},\text{Oxy}\right). \end{array}$$

This reward function gives a greater positive reward of 0.8 to both selfless and selfish agents if they satisfy their nature by adjusting the levels of their neurotransmitters.

Reward based on extrinsic motivation *R*_Ext_ whenever any agent dies, is given as follows:

(3) $$\begin{array}{c} R_{\text{Ext}}=-\left(\text{Remaining time of the simulation}*\text{discount factor}\right). \end{array}$$

Here discount factor is set to 0.1, which ensures that the reward stays within the range of [−1, 0]. This dynamic reward function makes sure to give a greater negative reward if an agent dies during the episode and less-negative reward if the agent dies near the end of the episode. *R*_Ext_ is given to every agent if an agent dies to motivate the agents for collective survival. The following equation gives the total accumulative reward.

(4) $$\begin{array}{c} R_{\text{Total}}=R_{\text{Int}}+R_{\text{Ext}}. \end{array}$$

#### 3.3.11. Emotional Brain

Deep Q-network (DQN), which is a method of deep reinforcement learning (DRL) [70], is used to develop the brain of every emotional agent because it is a continuous problem with no terminal state [71]. By interacting with the environment at discrete time steps (*t*=0,1,2…), emotional DRL agents learn different policies. Environment state space is denoted by *S* which consists of all the available information consisting of all the internal and external information of agents and the location of food reservoirs. Action space *A* consists of the possible actions an agent can perform, that is, *A*={No action, Up, Down, Left, Right, Eat, Share}. *R* represents the reward state. At every time step *t*, every agent observes a state *s*_*t*_ ∈ *S* and selects an action *a*_*t*_ ∈ *A*. In return, the agent gets a reward of *R*_Total_ ∈ *R* and moves to a new state *s*_*t*+1_=*S*. The agent's goal is to maximize the reward by finding the optimal policy *λ* : *S*⟶*A*, that is, the mapping of observed states and the action taken by the agent in those states.

To address the task as mentioned earlier of DRL, Q-learning is used. The choice of Q-function, the quality of state-action pair (*s*_*t*_, *a*_*t*_), is critical to the success of the Q-learning technique. Deep Q-network (DQN) uses deep neural network (DNN) to learn the Q-functions through iterative updates based on the experience. Neural network with one input layer, three hidden layers, and one output layer is used to approximate the action values *Q*=(*s*_*t*_, *a*_*t*_, *θ*), where *θ* represents the learning parameters of the neural network.

The network's input is the agent's state of the environment containing the information about the location of food reservoirs and other agents, food levels of agents, its neurotransmitter levels, and the current simulation time. The output is the approximate Q-value of every possible action that the agent can take as shown in Figure 5. The equation to calculate the Q-values is given as follows:

(5) $$\begin{array}{c} Q\left(s_{t},a_{t},\theta \right)=R_{\text{Total}}+\gamma {\text{max}}_{a_{t+1}}Q\left(s_{t+1},a_{t+1},\theta \right), \end{array}$$

where *R*_Total_ is the immediate reward that the agent gets on choosing the best action that gives the maximum Q-value of the next state represented by max_*a*_*t*+1__*Q*(*s*_*t*+1_, *a*_*t*+1_, *θ*). *γ* is the discount factor. The algorithm of temporal difference (TD) is used [72]. It enables the agent to update its knowledge on every timestep *t*. The formula is given as follows:

(6) $$\begin{array}{c} \text{TD}\left(a_{t},s_{t}\right)=R_{\text{Total}}+\gamma \;{\text{max}}_{a_{t+1}}Q\left(s_{t+1},a_{t+1},\theta \right)-Q\left(s_{t},a_{t},\theta \right). \end{array}$$

Substituting equation (6) in equation (5) makes the following equation:

(7) $$\begin{array}{c} Q\left(s_{t},a_{t},\theta \right)=Q\left(s_{t},a_{t},\theta \right)+\alpha \text{TD}\left(a_{t},s_{t}\right). \end{array}$$

DQN is to minimize the mean squared error of the temporal difference, which is shown above. *α* represents the learning rate.

## 4. Experimentation

This section explains the experimentation based on the proposed neurotransmitter-based deep Q-learning computational model. The simulation environment consists of four food reservoirs and two types of agents.

- Selfless agents
- Selfish agents

The grid world environment is developed in the Unity3D platform with the gird size of 10 × 10. Food reservoirs and agents are placed randomly in the environment. Each episode runs for 9 minutes, and after the completion of an episode, the environment resets. The environment also resets when all the agents die before the time of the episode runs out. Each experiment is trained for 100 episodes. DQN brain, implemented in python, is used for the training of the agents. Two experiments are done with altering the number of selfless and selfish agents and checking the effect on the survival time of the agents.

### 4.1. Food Reservoir

Each food reservoir is initialized with the available food level of 4 (Table 3), which is less than the total food needed by all agents for their survival. It ensures that the situation of social dilemma arises as depicted in Game Theory [73]. Both selfish and selfless agents can consume food from the reservoirs. It is done if the distance between the agent and a particular reservoir is less than 1, and the agent performs the action Eat. Otherwise, the action Eat has no effect.

Whenever the agent takes food from the reservoir, the food level of the agent is increased, and the reservoir storage is decreased. After every minute, the food in every reservoir is regenerated, and the available food is incremented by 0.5. Once the food level is less than 1 in a reservoir, it will not provide food to any agent.

### 4.2. Selfless and Selfish Agents

Agents are initialized with the food level of five. Following are the seven actions that selfless and selfish agents can perform {No Action, Up, Down, Left, Right, Share, and Eat}. After every minute, the food level of the agents gets decremented by 1. If the food level of any agent is less than 3, it is pushed in an FIFO (First In First Out) queue of needy agents. These are the agents whose food level is less than 3, and they need food from other agents. Both selfless and selfish agents transfer food to the first needy agent in the queue only if its food is greater than 3, as depicted by Maslow's hierarchy of needs [41]. When an agent performs the share action, its food level gets decremented by 0.5, and the food of needy agent (with whom the agent has shared) gets incremented by 0.5. The agent dies if the food level decreases to 0.

### 4.3. DQN Brain

The learning rate of the neural network used for the training of agents is set to 0.0001. Environmental states are passed to the network in batches of 32. The number of nodes in the input layer is 67. First, second, and third hidden layers contain 128, 128, and 64 nodes, respectively. The number of nodes in the output layer is 7. The memory size of each agent to remember the previous states and corresponding actions taken in those states is 100,000. The value of discount factor *γ* is 0.9.

### 4.4. Experiment 1

The first experiment (Figure 6) was conducted with eight virtual agents. All were initialized with a selfish personality having agreeableness and neuroticism value 0.2 and 0.8, respectively.

### 4.5. Experiment 2

The second experiment (Figure 7) was also conducted with eight virtual agents. Out of the eight agents, three agents were initialized with a selfish personality having agreeableness and neuroticism value 0.2 and 0.8, respectively, the same as the first experiment. The remaining five agents were initialized with the selfless personality having agreeableness and neuroticism 0.8 and 0.2, respectively.

## 5. Results

Table 4 shows the survival time of the agents collectively as a community for both the experiments.

Figures 8 and 9 show the Eat and Share actions performed by all the selfish agents during Experiment 1. The *x*-axis shows the no. of episodes, whereas the *y*-axis shows the total number of actions performed during a particular episode.

Figures 10 and 11 show the Eat and Share actions performed by all the selfless and selfish agents during Experiment 2. The *x*-axis shows the no. of episodes, whereas the *y*-axis shows the total number of actions performed during a particular episode.

Figures 12 and 13 show the Eat and Share actions performed by one selfish and one selfless agent during the 53rd episode of Experiment 2. The *x*-axis shows the time in seconds on which the specific action was performed. Whereas, *y*-axis and *z*-axis show the level of dopamine and oxytocin, respectively, at the particular time the specific action was performed.

## 6. Discussion

First research question addresses the concept of believability in virtual agents. Believability in virtual agents is based on the personality and emotions of the agents. Furthermore, there are five personality traits, according to the OCEAN Model. From those five traits, Agreeableness and Neuroticism are best suited for the situations of social dilemmas in virtual agents. These two personality traits made the agents selfish and selfless thus contributing to the believability in virtual agents. Moreover, the regulation of emotions according to the personality depends on the neurotransmitters. Dopamine and oxytocin are classified as selfish and selfless neurochemicals, respectively. In this work, we introduce two neurochemicals to introduce emotions and, subsequently, believability.

We performed two experiments to evaluate whether the proposed method introduces believability and how effective it is to solve the social dilemma problems. In the first experiment, all eight agents were selfish, whereas, in the second experiment, five agents were selfless, and three were selfish. Agents were given seven actions {No action, Up, Down, Left, Right, Eat, and Share}. On performing any of those actions, their neurochemicals change. It is evident from Figures 8 and 9 of the first experiment and Figures 10 and 11 of the second experiment that selfish agents performed more eat actions and fewer share actions to keep their dopamine level high and oxytocin level low (Figures 12 and 13). However, selfless agents performed more share actions to keep their oxytocin level high (Figure 13). Agents chose those actions that maintained their neurotransmitters in the desired range according to their personality. Therefore, it was concluded that we can introduce believability in virtual agents by regulating the emotions through neurotransmitters according to the agents' personality with the reinforcement learning technique.

Second research question investigates the effect of emotions on cooperation between agents. In the situation of social dilemmas with limited resources, the situation worsens if people behave selfishly. When people keep their benefits aside and cooperate selflessly, the situation becomes relatively favorable. Therefore, we believed that if we introduce agents with empathetic and selfless personality in the virtual social dilemma situation, the cooperation between the agents can be increased. We also measured the total time for which all the agents were alive (Table 4) while food resources kept the same in both experiments. In Experiment 1, selfish agents ate food for themselves and shared less food with others. Therefore, they could survive collectively for 6 minutes and 10 seconds only (Table 4). However, in Experiment 2, selfless agents ate food from the reservoir and shared food with the needy agents. Therefore, the survival time was increased to 7 minutes and 55 seconds (Table 4). All agents in Experiment 2 survived for 1 minute and 45 seconds more than the eight selfish agents in Experiment 1 with the same food resources.

Hence, it proved that when we increase the number of selfless agents with a high agreeableness personality trait, they started cooperating with others by regulating their positive emotions through neurotransmitters according to their personality. Thus, the situation of social dilemmas improved.

Third research question measures the effect of emotions by controlling virtual neurotransmitters on the decision-making capability of agents. Reinforcement learning is a continuous learning process in which the problem is modeled as Markov decision process (MDP). In our reinforcement learning-based approach, an agent utilizes its previous experience (actions taken in the past) to improve the decisions in the future. The agent with the passage of time discovers which actions give the maximum reward by exploiting and exploring them. Thus, the agent starts to take actions whom Q-values are greater. In our experimentations about reward maximization, selfish agents learnt not to share the food whereas selfless agents learnt to share food with needy agents (who were unable to eat from the reservoir due to limited food) as the training episodes passed. Therefore, through reinforcement learning, agents learnt to keep their neurotransmitters in the desired range according to their personality. Thus, agents were achieving the maximum reward by performing the specific actions that best suited their personality without being explicitly told. This shows that the decision-making capability of agents was improved under reinforcement learning.

In the experiments, we measured the total time for which all the agents were alive (Table 4) while food resources kept the same in both experiments. In Experiment 1, selfish agents ate food for themselves, as shown in Figure 8. The number of eat actions performed collectively by selfish agents are greater (Figure 8) than the number of share actions (Figure 9). Due to limited food available in the reservoirs, agents were able to survive collectively for 6 minutes and 10 seconds only (Table 4) after 100 episodes of training. After 6 minutes and 10 seconds, first agent died in the environment. However, in Experiment 2, selfless agents ate food from the reservoir as shown in Figure 10. After eating the food, selfless agents also shared the food with the needy agents. It is evident that the number of Share actions in Experiment 2 (Figure 11) is greater than the Share actions performed in Experiment 1 (Figure 9). The survival time was increased to 7 minutes and 55 seconds (Table 4) in this case. All agents in Experiment 2 were able to survive for 1 minute and 45 seconds more than the eight selfish agents in Experiment 1 with the same food resources. It proved that when we increase the number of selfless agents with a high agreeableness personality trait, they started to perform more share actions thus cooperating with others agent. This was because, the selfless agents tried to maximize their reward by regulating their positive emotions through neurotransmitters according to their personality. In return, the situation of social dilemma was improved.

Therefore, we hypothesized that we can introduce emotions by controlling and regulating the virtual neurotransmitters in agents through the reinforcement learning technique to increase the decision-making capability of the agents according to their personality. Two experiments were conducted with varying the number of selfless and selfish agents to evaluate the solution. Both types of agents tried to maximize their reward function by performing actions with the highest Q-value (8). For selfish agents, dopamine level greater than 2 and oxytocin level lower than 4 acquire maximum reward. According to (8), Q-value for Eat action was mostly greater than Share action. Therefore, selfish agents performed more Eat actions for increasing their dopamine level (Figure 12).

Moreover, they avoided sharing food, which resulted in the oxytocin level having a small value (Figure 13). Similar to selfish agents, selfless agents in the second experiment also tried to maximize their reward function. But for selfless agents, maximum reward requires higher dopamine, that is, greater than 4 and higher oxytocin level, that is, greater than 5. Selfless agents tried to keep their dopamine and oxytocin levels high by consuming the food and then sharing it with the needy agents. In each episode, the Q-value of the action Eat was greater for the first 3 minutes; therefore, both selfish and selfless agents consumed food from the reservoir (Figure 12). After 3 minutes, the Q-value of the action Share was greater for the selfless agents only (Figure 13). Agents can share the food only when their food level is greater than 3. To maximize the reward, selfless agents shared food with needy agents (who could not eat from the reservoir due to limited food).

Therefore, agents learned to keep their neurotransmitters in the desired range through reinforcement learning according to their personality. Thus, achieving the maximum reward by performing the specific actions that best suited their personality. Hence, their decision-making capability was improved.

## 7. Conclusion

To solve the situation of social dilemmas in virtual agents, we proposed a neurotransmitter-based deep Q-learning model for emotional modeling in agents. Agents maintained their neurotransmitter levels by performing specific actions that maximize intrinsic and extrinsic rewards according to their personality. This mapping of actions to neurotransmitters improved the decision-making capability of the agents and developed cooperation between the agents. Experiments showed that selfless agents cooperated with one another, and they survived the social dilemma situation for 1 minute and 45 seconds more than selfish agents. We have concluded that the agents' personality and their emotion regulation through neurotransmitters introduced believability in virtual agents, and selfless agents, in the environment, helped to avoid social dilemma problems that improved the overall survival of the community.

This work opens up a new dimension for emotion modeling in virtual agents. We have chosen a complex social dilemma scenario to see how agents behave in a comparatively large environment. For application point of view, this work can be used for developing nonplayer characters (NPCs) in games. Future directions for extending this research can include extending the experiments using all the four neurotransmitters. Second, we can devise methods that will evolve the personalities of the agents according to the environmental changes.

## Figures and Tables

**Figure 1:** Solving social dilemma situation by introducing believability through personality and neurotransmitters in virtual agents.

**Figure 2:** Architecture diagram of the neurotransmitter-based deep Q-learning emotional model with reward calculation based on intrinsic and extrinsic motivation of the emotional agent.

**Figure 3:** Ocean model of personality.

**Figure 4:** Four types of neurotransmitters.

**Figure 5:** Neural Network used for Q-Learning.

**Figure 6:** Grid world Unity3D image taken during the training of the first experiment. Plus signs in green show the food reservoirs and red cubes show the selfish agents.

**Figure 7:** Grid world Unity3D image taken during the training of the second experiment. Plus signs in green show the food reservoirs, red cubes show the selfish agents, and white cubes show the selfless agents.

**Figure 8:** Cumulative Eat actions of eight selfish agents during 100 episodes of first experiment.

**Figure 9:** Cumulative Share actions of eight selfish agents during 100 episodes of first experiment.

**Figure 10:** Cumulative Eat actions of five selfless and three selfish agents during 100 episodes of second experiment.

**Figure 11:** Cumulative Share actions of five selfless and three selfish agents during 100 episodes of second experiment.

**Figure 12:** Changes in neurotransmitters of one Selfless and one Selfish agent during the 53rd episode of the second experiment while performing eat action.

**Figure 13:** Changes in neurotransmitters of one Selfless and one Selfish agent during the 53rd episode of the second experiment while performing share action.

**Table 1:** Research matrix for comparison of related works.

Research work	Reinforcement learning	Social dilemma in MAS	Emotions in social dilemmas	Cooperation
Bates [40, 41]	✘	✘	✘	✘
Sloman [43, 44]	✘	✘	✘	✘
Blumberg [45], El-Nasr et al. [34, 49]	✘	✘	✘ (Emotional virtual pets)	✘
Silverman et al. [50–52]	✘	✘	✘ (Human behavioral models in game engines)	✘
Huang et.al [59]	✔	✔ (Only for two agents)	✘	✔
Diallo et al. [55]	✔	✘	✘	✔
Leibo et al. [11]	✔	✔ (Only for two agents)	✘	✔
Broekens et al. [56]	✔	✘	✘	✘
Sequeira et al. [57]	✔	✘	✘	✘
Our proposed model	✔	✔	✔	✔

**Table 2:** Values of personality traits for both selfless and selfish agents.

Sr. no.	Personality of agent	Agreeableness	Neuroticism
1	Selfless	0.8	0.2
2	Selfish	0.2	0.8

**Table 3:** The initial levels of neurotransmitters and the food level of both types of agents at the beginning of the experiments.

Agents	Food level	Dopamine	Oxytocin	Agreeableness	Neuroticism
Selfless	5	1	4	0.8	0.2
Selfish	5	1	2	0.2	0.8

**Table 4:** Collective survival time of the agents for both experiments.

Sr. no.	Time of collective survival (hh:mm:ss)
Experiment 1 (eight selfish agents)	00:06:10
Experiment 2 (five selfless and three selfish agents)	00:07:55

## Data Availability

No data were used to support this study.
